This article has been retracted.

# Disruption of Growth Hormone Receptor Prevents Calorie Restriction from Improving Insulin Action and Longevity

**DOI:** 10.1371/journal.pone.0004567

**Published:** 2009-02-23

**Authors:** Michael S. Bonkowski, Fernando P. Dominici, Oge Arum, Juliana S. Rocha, Khalid A. Al Regaiey, Reyhan Westbrook, Adam Spong, Jacob Panici, Michal M. Masternak, John J. Kopchick, Andrzej Bartke

**Affiliations:** 1 Department of Internal Medicine – Geriatrics Research, Southern Illinois University School of Medicine, Springfield, Illinois, United States of America; 2 Department of Pharmacology, and Physiology, Southern Illinois University School of Medicine, Springfield, Illinois, United States of America; 3 Instituto de Química y Fisicoquímica Biológicas (IQUIFIB), Facultad de Farmacia y Bioquímica, Universidad de Buenos Aires, Buenos Aires, Argentina; 4 Department of Morphology, Laboratory of Cellular Biology, Institute of Biological Sciences, Federal University of Minas Gerais, Belo Horizonte, Brazil; 5 Department of Physiology, College of Medicine, King Saud University, Riyadh, Saudi Arabia; 6 Department of Biomedical Sciences, Edison Biotechnology Institute, Ohio University, Athens, Ohio, United States of America; University of Bremen, Germany

## Abstract

Most mutations that delay aging and prolong lifespan in the mouse are related to somatotropic and/or insulin signaling. Calorie restriction (CR) is the only intervention that reliably increases mouse longevity. There is considerable phenotypic overlap between long-lived mutant mice and normal mice on chronic CR. Therefore, we investigated the interactive effects of CR and targeted disruption or knock out of the growth hormone receptor (GHRKO) in mice on longevity and the insulin signaling cascade. Every other day feeding corresponds to a mild (i.e. 15%) CR which increased median lifespan in normal mice but not in GHRKO mice corroborating our previous findings on the effects of moderate (30%) CR on the longevity of these animals. To determine why insulin sensitivity improves in normal but not GHRKO mice in response to 30% CR, we conducted insulin stimulation experiments after one year of CR. In normal mice, CR increased the insulin stimulated activation of the insulin signaling cascade (IR/IRS/PI3K/AKT) in liver and muscle. Livers of GHRKO mice responded to insulin by increased activation of the early steps of insulin signaling, which was dissipated by altered PI3K subunit abundance which putatively inhibited AKT activation. In the muscle of GHRKO mice, there was elevated downstream activation of the insulin signaling cascade (IRS/PI3K/AKT) in the absence of elevated IR activation. Further, we found a major reduction of inhibitory Ser phosphorylation of IRS-1 seen exclusively in GHRKO muscle which may underpin their elevated insulin sensitivity. Chronic CR failed to further modify the alterations in insulin signaling in GHRKO mice as compared to normal mice, likely explaining or contributing to the absence of CR effects on insulin sensitivity and longevity in these long-lived mice.

## Introduction

A vast majority of the mutations that delay aging and prolong lifespan in the mouse (*Mus musculus*) either directly or indirectly alter somatotropic and/or insulin signaling [1], [2]. There is considerable intra- and extra-cellular crosstalk between growth hormone (GH), insulin-like growth factor 1 (IGF-1), and insulin in mediating growth and metabolism in mammals [3]. These signaling pathways are highly conserved across phyla; and mutations affecting homologous IGF-1/insulin-like signaling and downstream gene expression increase longevity in yeast (*Saccharomyces cerevisiae*), worms (*Caenorhabditis elegans*), and flies (*Drosophila melanogaster*) [4], [5]. Taken together, the above-mentioned findings posit GH/IGF-1/insulin (and homologous) signaling as one of the key mediators of longevity.

Calorie restriction (CR) is the only environmental treatment known to consistently increase average and maximal lifespan and delay aging in organisms ranging from yeast to mammals [6], [7]. In addition to extended longevity and reduced cancer incidence, the most consistent responses to CR in mammals include reductions in peripheral (i.e. blood) insulin, GH, IGF-1, and glucose levels [6], [8]. These biomarkers of a “CR response” are reported in species ranging from mice to humans [4]. Interestingly, there is considerable phenotypic overlap between mice on CR and many long-lived mutant mice. These similarities include reductions in body weight, body size, neoplastic disease incidence, peripheral GH/IGF1, insulin, and glucose, relative to their respective controls [9]–[11]. In addition, most of the long-lived mutant mice and mice on long-term CR show improvements in insulin sensitivity, feed efficiency and health-span. These similarities suggest that studying interactions between the life-extending mutations and CR may reveal what pathways and mechanisms are utilized by CR to alter aging.

GH receptor/binding protein knockout (GHRKO) mice were developed by targeted disruption of the GHR/GHBP gene [12]. This insertion mutation renders the GH receptor nonfunctional and causes severe GH resistance, leading to suppression of peripheral IGF-1 and insulin levels. In addition, GHRKO mice are markedly insulin-sensitive, tend to be hypoglycemic, have reduced body weight and size, reduced incidence of neoplastic disease and a pronounced increase in all lifespan parameters, including increased mortality rate doubling time (MRDT), as well as median, average and maximal lifespan [10], [13], [14]. We previously reported that in contrast to hypopituitary, GH-deficient Ames dwarf mice [15], GHRKO mice did not receive a CR benefit in insulin sensitivity and most measures of longevity [16]. From a genetic perspective, these findings suggest that CR may work partially via GH signaling to mediate improvements in insulin sensitivity and extended lifespan, especially since it is well known that GH can induce insulin resistance [17]–[19]. One possible caveat is that when using a single level of CR, it is difficult to conclude whether the mutation ablates the effects of CR at all “doses” (*i.e.*, flat-lines the dose-response curve) or if the mutation altered (or shifted) the CR dose response curve [20]. While both outcomes are important, the former would implicate GHR-based signaling as the paramount pathway controlling the effects of CR on aging and lifespan in mice and thus potentially one of the pathways that may be exploited to induce CR-like effects in humans.

We report here two long-term studies, of the interaction between GHR disruption and CR in male mice that were designed to address the following questions: 1) Does the GHRKO mutation modulate or completely ablate the benefits of CR on lifespan? 2) How does CR improve insulin sensitivity and longevity in normal mice? 3) Why does CR fail to improve insulin sensitivity and longevity in GHRKO mice?

## Results and Discussion

### Longevity characteristics of normal and GHRKO mice on mild CR

To determine whether the previously documented differential responses of GHRKO and normal (N) mice to 30% CR may have been limited to this level of dietary restriction, we conducted an additional longevity study using a milder degree of CR in both mice. Every other day (EOD) feeding resulted in approximately a 10–15% reduction in the average daily food intake compared to *ad libitum* (AL) control mice (data not shown) [21], [22]. In normal male mice, EOD feeding led to a 16% increase in median lifespan (N AL = 851 days vs. N EOD = 1010 days, hazard ratio (HR) 2.62 confidence interval (CI) 1.31–6.03). In contrast, median lifespan of GHRKO mice was not extended (KO AL = 1178 days vs. KO EOD = 1158 days, HR 1.063, CI 0.50–2.29). Compared to N AL mice, EOD feeding increased overall lifespan in normal mice as evaluated by log-rank analysis (P<0.008); however, there were no significant diet effects in GHRKO mice (P = 0.6727). Thus, a milder and different form of CR that increased longevity in normal control mice failed to further increase the lifespan of long-lived GHRKO mice, corroborating our previous findings using a more severe (30%) traditional CR regimen [16]. Taken together, these studies indicate that GH resistance ablates rather than modulates (or shifts) the benefits of CR on longevity in male GHRKO mice.

### Effects of long-term 30% CR on metabolic characteristics of normal and GHRKO mice

To search for potential mechanisms for the differential responses of GHRKO and normal mice to CR and to further investigate the interaction between CR, GH resistance and insulin sensitivity, 30% CR was initiated at 2 months of age and maintained for one year in normal and GHRKO male mice. In comparison to animals fed AL, CR produced the expected decrease in body weight trajectory in both normal and GHRKO mice (Figure 1A). Furthermore, we fasted mice in all groups overnight to determine body weight in the non-fed state. Compared to AL controls, one year of 30% CR led to reduced fasted body weight in both normal and GHRKO mice (Figure 1B). There were no significant differences in the fasted peripheral glucose levels in any of the groups tested (Figure 1C). In normal mice, CR decreased the level of fasted insulin (P<0.001), while both AL and CR GHRKO mice had reduced insulin levels compared to normal mice on either diet (P<0.001 for each comparison). Calorie restriction did not further decrease fasted peripheral insulin levels in GHRKO mice (Figure 1D).

**Figure 1:** Metabolic parameters of male GHRKO (KO) and normal (N) mice fed *ad libitum* (AL) or subjected to 30% calorie restriction (CR) for one year. Panel (A) shows time-course changes in body weight over a one year period. After one year of CR, all groups were fasted overnight and bodyweight (B), peripheral glucose (C), insulin (D), and calculated homeostatic model of assessment (HOMA, E) were determined. Values with unlike superscripts/letters are significantly different (P<0.05).

The relationship between peripheral glucose and insulin levels is an important indicator of the overall insulin sensitivity of the animal. One model that utilizes fasted glucose and insulin levels to represent the whole organism's insulin sensitivity is the Homeostatic Model of Assessment (HOMA), with a relatively lower score representing improved insulin sensitivity. Figure 1E shows that in normal mice, one year of CR led to a reduction in the HOMA score compared to AL controls (P<0.01), while CR did not alter the already improved HOMA score in GHRKO mice.

To summarize, CR reduced body weight in both phenotypes and improved fasting insulin sensitivity in normal mice, but failed to further improve the already insulin-sensitive status of GHRKO mice, thus uncoupling the effects of CR on body weight/growth from its effects on insulin sensitivity and lifespan. To further explore the interaction between GH resistance, CR, and insulin sensitivity, we investigated the activation state of the insulin signaling cascade in these groups in response to an exogenous insulin challenge.

### Effects of CR on the response of normal and GHRKO mice to insulin stimulation

The actions of insulin are critical for the regulation of the processes involved in glucose homeostasis. The maintenance of carbohydrate homeostasis involves multiple enzymatic processes, in addition to cellular signaling processes, with liver and muscle playing different roles. To determine the molecular mechanism of differential impact of CR on insulin sensitivity in normal mice and GHRKO mice, we evaluated insulin signal transduction through the IR/IRS/PI3K/AKT1/AKT2 pathway in liver and skeletal muscle in normal and GHRKO mice fed AL or subjected to CR for one year in response to an insulin challenge (10 IU/kg insulin versus saline).

### Liver responses to insulin stimulation

Calorie restriction increased total amount of insulin receptor (IR) protein in normal mice (P<0.03), but did not increase the already-elevated levels of IR in GHRKO mice on both AL and CR diets (Figure 2A). The heightened insulin induced upstream events in GHRKO mice corresponds with previous studies in these insulin sensitive mutants [23], [24]. In response to acute insulin stimulation, normal mice on CR had a 2-fold greater increase in IR activation (as estimated by measuring IR phosphorylation at tyrosine (Tyr) residue 1158 [pY1158] as a proxy for activation) than the normal AL mice, while CR did not increase the already elevated insulin-induced IR activation in GHRKO mice (Figure 2B).

**Figure 2:** Liver insulin signaling cascade total proteins and phospho-proteins in response to insulin stimulation (10 IU/kg) versus saline treated controls in GHRKO (KO) and normal (N) mice fed *ad libitum* (AL) or 30% calorie restricted (CR) for one year. ELISA with antibodies directed towards total insulin receptor (IR; A), IR pY1158 (B), AKT1 (D), and AKT1 pS473 (E) were performed. Liver homogenates were immunoprecipitated (IP) with anti-p85, separated using SDS-PAGE and the level of non-specific Tyr phosphorylation was determined at approximately 180 kDa using anti-pY99 (C). Total AKT2 protein (F) and AKT2 pS473/474 (G) was determined from liver protein homogenates first subjected to IP using anti-AKT2. Panel (H) summarizes key insulin-stimulated phospho-proteins compared to insulin-stimulated N AL mice. Bands are representative blots from 4–6 male mice per phenotype/diet/treatment group. Values with unlike superscripts/letters are significantly different (P<0.05).

Next, we determined the levels of activation of a major intracellular signaling intermediate in the insulin signaling cascade, namely phosphatidylinositol-3 kinase (PI3K). In normal mice, CR significantly increased insulin-induced p85/IRS pY99 phosphorylation from 1.8-fold (N AL) to 2.2-fold in (N CR). However, this parameter was not affected by CR in GHRKO mice (Figure 2C). This finding suggests that while the enhanced amplitude of the insulin signal from the hepatic IR was maintained at the level of PI3K in normal mice on CR, GHRKO mice on either diet did not show the level of activation (as presumed by phosphorylation) that corresponded to the upstream activation of the insulin receptor (Figure 2B).

An important downstream target of the insulin/PI3K signaling cascade is protein kinase B (AKT1). Total AKT1 protein in liver did not differ in any of the groups tested (Figure 2D). In normal mice, CR increased the insulin-induced phosphorylation of AKT1 at serine (Ser) residue 473 (pS473, a marker of activation of this enzyme) compared to values measured in insulin-stimulated N AL mice (P<0.03, Figure 2E). Insulin-induced pS473 levels of AKT in KO AL and KO CR groups did not significantly differ from the corresponding values in N AL or N CR mice.

In the liver of normal mice, CR increased AKT2 total protein compared to AL controls (P<0.03, Figure 2F). GHRKO mice had comparable AKT2 total protein levels when compared to N AL mice. Acute insulin stimulation increased the levels of Ser phosphorylated AKT2 (pS474) in all groups (P<0.001). When compared to phenotype/treatment saline controls within groups, insulin increased the phosphorylation in N AL by 92%, while N CR, KO AL, and KO CR groups had more than a 2 fold increase in insulin stimulated phosphorylation (N CR 2.1 fold, KO AL 2.05 fold, and KO CR 2.1 fold).

Hepatic insulin signaling cascade activation in response to insulin stimulation in normal mice on CR and in GHRKO mice on both diets is compared to N AL controls and summarized in Figure 2H. These data suggest that CR increases the levels of proteins involved in insulin signaling transduction and the activation of these proteins in response to insulin in normal mice, but has no effects in GHRKO mice. Curiously, the enhanced activation of the IR in response to insulin stimulation is not propagated downstream to the AKT proteins in GHRKO mice, whereas it is in the normal mice. In an attempt to understand this discrepancy, we explored the regulatory subunits of PI3K in normal and GHRKO mice fed AL or subjected to 30% CR.

### Determination of the PI3K regulatory subunits p85/p55/p50

To determine the relative protein abundance of the regulatory subunits of PI3K in the liver, we targeted the p85 subunit of PI3K for immunoprecipitation in liver homogenates and subsequently immunoblotted for the p85, p55 and p50 subunits of PI3K (Figure 3). In the liver of normal mice, CR did not alter p85 (Figure 3A), p55 (Figure 3B) or p50 (Figure 3C) total protein concentration. Similar to these findings, CR did not alter the level of these subunits in GHRKO mice, with the exception of a significant reduction in the p55 subunit compared to GHRKO AL controls (P<0.05). It has been shown that an alteration in a single regulatory subunit of PI3K may act to inhibit or bind up free IRS proteins and alter signal transduction [25], [26]. This could explain the partial decrease in signal amplification seen between the activation of the IR and PI3K phosphorylation in mice from the normal CR group. Irrespective of the diet, GHRKO mice had reduced p85, p55, and p50 regulatory subunits compared to normal mice. CR did reduce the p55α subunit in GHRKO mice. We believe this reduction of the regulatory subunits of PI3K in GHRKO mice may underpin the dampened downstream activation (compared to activation of IR) of the PI3K/IRS, AKT1 and AKT2 proteins seen in the insulin stimulation experiments (Figures 2 and 3).

**Figure 3:** Liver PI3K subunit abundance in GHRKO (KO) and normal (N) mice fed *ad libitum* (AL) or 30% calorie restriction (CR) for one year. Liver protein isolates were immunoprecipitated (IP) with anti-pan-p85. Total p85α (A), 55α (B) and 50α (C) subunits were separated using SDS-PAGE, transferred to nitrocellulose membranes and blotted with anti-pan-p85. Bands are representative blots from 4–6 male mice per phenotype/diet/treatment group. Values with unlike superscripts/letters are significantly different (P<0.05).

### Effects of insulin stimulation in the skeletal muscle

Skeletal muscle is the major site of insulin-stimulated glucose uptake in the body, as demonstrated by various tissue-specific knockouts of the glucose transporter GLUT4 [27]. In normal mice, CR increased total IR from 6.92±0.64 to 8.87±0.47 units/100ug (P<0.02, Figure 4A). In contrast, GHRKO AL mice had elevated muscle IR protein that was reduced by CR (9.01±0.90 to 6.72±0.59 units/100ug; P<0.01). Insulin-stimulated phosphorylation of the IR in normal CR mice was increased approximately 3-fold compared to AL controls (P<0.001), while IR phosphorylation in GHRKO mice was unaffected by the diet, and values obtained were comparable to normal AL mice (Figure 4B). This finding was also reported previously [24], and this does not correspond with their heightened insulin stimulated glucose uptake [16] so we therefore further investigated downstream insulin signaling events associated with insulin mediated glucose uptake.

**Figure 4:** Muscle insulin signaling cascade total proteins and phospho-proteins in response to insulin stimulation (10 IU/kg) versus saline treated controls in GHRKO (KO) and normal (N) mice fed *ad libitum* (AL) or 30% calorie restriction (CR) for one year. Levels of total insulin receptor (IR; A), IR pY1158 (B), AKT1 (D), and AKT1 pS473 (E) were determined using ELISA. Liver homogenates were immunoprecipitated (IP) with anti-p85, separated using SDS-PAGE and the level of non-specific Tyr phosphorylation was determined at approximately 180 kDa (corresponding to IRS proteins) using anti-pY99 (C). Total AKT2 protein (F) and AKT2 pS473/474 (G) was determined from liver protein homogenates first subjected to IP using anti-AKT2. Total GLUT4 protein (H) was determined in muscle homogenates using anti-GLUT4. Panel (I) summarizes key insulin-stimulated phospho-proteins compared to insulin-stimulated N AL mice. Bands are representative blots from 4–6 male mice per phenotype/diet/treatment group. Values with unlike superscripts/letters are significantly different (P<0.05).

Calorie restriction produced a significant increase in the PI3K/IRS phosphorylation of IRS associated with PI3K in the muscle of normal mice, yet did not further elevate the already heightened phospho-Tyr levels in the GHRKO mice (Figure 4C). This finding did not coincide with IR activation, where GHRKO mice did not show elevations in IR phosphoylation, yet there was an increase in the level of IRS phosphorylation at Tyr 99. To further probe this finding, we assessed the total protein and phosphor-Ser levels of the downstream targets AKT1, AKT2, and mTOR, as well as the total protein content of GLUT4.

AKT proteins in skeletal muscle are critically involved in insulin-stimulated glucose uptake through the trafficking of GLUT4 to the cell surface. In normal mice, CR increased total AKT1 protein (N AL 11.2±0.94 versus N CR 16.4±2.0, P<0.01, Figure 4D). In contrast, CR did not increase the already-elevated level of AKT1 total protein in GHRKO mice. Calorie restriction increased insulin-induced AKT1 phosphorylation in normal mice (P<0.01), but it did not further increase the already-elevated AKT1 response to insulin in GHRKO mice (Figure 4E). This data coincide with the increases of p85/IRS activation in muscle homogenates shown in Figure 4C.

As mentioned previously, AKT2 has been shown to mediate the stimulatory effects of CR on improved glucose uptake in skeletal muscle [27]. Calorie restriction did not alter muscle AKT2 protein abundance in either phenotype, but total AKT2 protein was elevated in GHRKO AL mice compared to normal AL controls (P<0.05, Figure 4F). It should be noted that normal CR mice had numerically elevated AKT2 values (compared to normal AL mice) that were not significantly different from the elevated values in GHRKO groups. Calorie restriction increased AKT2 phosphorylation in response to insulin stimulation in normal mice, compared to insulin-stimulated AL controls (P<0.01), while GHRKO mice had elevated phosphor-Ser 474 AKT2 levels (P<0.01 for both, Figure 4G), with no further changes in response to CR. The similarity of activated AKT1 and AKT2 between normal mice on CR and GHRKO mice on either diet coincides with the improved insulin sensitivity in these groups compared to normal AL controls, and with our previous results concerning CR effects on longevity [16]. Since the AKT proteins have been shown to regulate insulin-stimulated GLUT4 trafficking, we next determined the level of GLUT4 protein in skeletal muscle whole cell homogenates.

Muscle GLUT4 total protein levels were significantly increased by CR in normal mice (P<0.003, Figure 4H). However, CR did not alter total protein levels in GHRKO mice. Both KO AL and KO CR mice had elevated muscle GLUT4 total protein levels compared to N AL controls (P<0.03 and P<0.04, respectively). These findings indicate that normal mice on CR and GHRKO mice on both diets have increased pools of GLUT4 available for recruitment. Figure 4I illustrates/summarizes the insulin signaling activation state of normal mice on CR and GHRKO mice (on both diets) compared to normal AL controls. GHRKO mice did not have elevated IR activation in comparison to their normal littermates, yet downstream PI3K/IRS-1, AKT1, AKT2 and GLUT4 levels or activity were elevated. While CR increased the activation of all proteins tested in normal animals, when compared to AL controls, the effects of CR in GHRKO mice were absent or opposite to those found in normal mice on CR. To further investigate this incongruity, we more closely examined the level of inhibition between the IR and PI3K signaling molecules.

### Calorie restriction and/or GH resistance decreases mTOR signaling and phosphoSer inhibition of IRS-1 in skeletal muscle

A number of recent reports show that Ser/Thr kinases mTOR, JNK, and PKCζ mediate a negative feedback loop in the insulin signaling cascade by phosphorylating IRS-1 at Ser position 307 [28], [29]. While IRS proteins are normally Tyr-phosphorylated upon IR activation, Ser phosphorylation prevents binding to the beta subunit of the IR and subsequent Tyr phosphorylation, thereby preventing the progression of insulin signal transduction. Since we have previously reported a reduction in JNK activation and in PKCζ in the skeletal muscle of GHRKO mice [30], we investigated the levels of IRS-1 total protein and phospho-Ser307 IRS-1 in normal and GHRKO mice on both dietary regimens. Total IRS-1 protein levels were not different in any of the groups tested (Figure 5A). Compared to normal mice, GHRKO mice had more than a 50% reduction in the phosphorylation of IRS-1 at Ser 307 (Figure 5B). We believe that the decrease in IRS-1 phosphorylation at this inhibitory site (Ser 307) in GHRKO mice underpins the insulin-stimulated elevations in the activation of downstream PI3K/IRS, AKT1 and AKT2 in the absence of increased IR activation upstream.

**Figure 5:** Muscle total IRS-1 protein (A) and IRS-1 pS307 inhibitory phosphorylation (B) in GHRKO (KO) and normal (N) mice fed *ad libitum* (AL) or 30% calorie restriction (CR) for one year was determined using ELISA. Bars represent 6–8 animals per phenotype/diet group. Values with unlike superscripts/letters are significantly different (P<0.05).

It was recently reported in another long-lived, insulin-sensitive mouse, the Ames dwarf, that mTOR signaling was reduced in skeletal muscle [30]. Since mTOR has been directly implicated in mediating IRS-1 inhibition through phosphorylation at Ser 307, we determined the level of mTOR total protein and its phosphorylated isoform in normal and GHRKO mice on both diets. In normal mice, CR reduced total mTOR protein compared to AL controls (P<0.01), while CR did not further reduce the already low levels of mTOR in GHRKO mice (Figure 6A). The activation of mTOR through phosphorylation at Ser 2448 followed the same trends as total content of mTOR protein, where CR reduced basal activation (pS2448) of mTOR in normal mice but did not alter the already low levels of activation in GHRKO mice (Figure 6B). We believe that differences in mTOR signaling implied by these results together with reduced JNK and PKCζ activation previously reported by our laboratory [31] importantly contribute to, and perhaps account for, the decrease in skeletal muscle inhibitory IRS-1 Ser 307 phosphorylation and improved muscle and whole-animal insulin sensitivity in GHRKO mice.

**Figure 6:** Muscle total mTOR protein (A) and mTOR pS2448 (B) in GHRKO (KO) and normal (N) mice fed *ad libitum* (AL) or 30% calorie restriction (CR) for one year were determined using western blotting. Bars represent 6–8 animals per phenotype/diet group.

### Conclusion

In the present study, we addressed three major research questions: 1) Does the GHRKO mutation modulate, or ablate, the effects of different intensities of CR on longevity? 2) How does CR improve insulin sensitivity and longevity in normal mice? and 3)Why does CR fail to improve insulin sensitivity and longevity in GHRKO mice?

In regard to the first question, we showed that while longevity of normal mice increased as expected in response to various intensities of CR, GHRKO mice did not derive longevity benefits from identical dietary interventions. This “flattening” of the median lifespan response in GHRKO mice on various levels of food intake shows that, in the absence of a functional GH receptor, CR does not affect longevity of male GHRKO mice. In other words, GH resistance ablates, rather than modulates, the key benefit of CR in these animals. In yeast and invertebrates the interactions between CR (or dietary restriction) and mutations that extend longevity have been explored [reviewed in 32]. While there seems to be homologous insulin signaling pathway mutations that ablate the CR response in yeast [i.e. Sch9, an AKT homologous protein and TOR, 33], mutations in chico (IRS-1 homologous proteins) modulate, rather than block, the CR response in flies [34]. These findings in less complex organisms are confounded by two major complications. First, yeast and invertebrates have not evolved GH signaling pathways. This fact makes it difficult to interpret findings across species. Second, the method by which dietary restriction, or CR is delivered in yeast and invertebrates is quite different than the traditional mammalian model, further complicating interaction studies [32].

In normal mice on CR, there is a major amplification of the insulin signaling cascade, with increases in protein concentration and/or (insulin-stimulated) activation of almost all the cellular mediators of insulin action tested in the present study (summarized in Figure 7). These increases in the insulin signaling cascade in liver and muscle show that the previously documented improvements in whole-animal insulin sensitivity in response to CR reflect heightened insulin cascade action. We previously postulated that improved whole-animal insulin sensitivity is tightly coupled to extended longevity [16].

**Figure 7:** Summarizes the effects of CR, or lack thereof, in wildtype and GHRKO mice under insulin-stimulated conditions. Solid grey proteins represent stimulatory activation, while solid black proteins are inhibitory.

The present results suggest two different—but not necessarily mutually exclusive—answers to our third question: “Why does CR fail to increase insulin sensitivity and longevity in GHRKO mice?” Since skeletal muscle is the major mediator of post-prandial, insulin-stimulated glucose uptake, we believe our data showing heightened muscle insulin action in both normal mice on CR and GHRKO mice regardless of diet underpin their improved insulin sensitivity (summarized in Figure 7). This convergence between normal mice exposed to long-term CR and innately insulin-sensitive GHRKO mice could explain why CR fails to further improve insulin sensitivity of GHRKO mutants or further extend their already-long lives. Another conclusion can be drawn from the differential effects of CR on the responses to an insulin challenge in the liver's insulin signaling cascade. While normal mice on CR showed improved downstream insulin action through increases in total protein and/or insulin-stimulated activation of several key elements of the insulin signaling cascade in liver, CR failed to produce corresponding changes in GHRKO mice. Additionally, both KO AL and CR groups had reduced downstream insulin-induced activation. This tissue-specific phenotypic dimorphism may have contributed to the absence of CR effects on whole-animal insulin sensitivity and lifespan in GHRKO mice.

Collectively, the present study identifies molecular steps of insulin signaling in the liver and in the muscle that are similarly affected by two conditions that extend life, CR in normal animals and deletion of the GH receptor, but are not altered by CR in GHRKO mice in which CR fails to increase insulin sensitivity and therefore longevity. This includes four parameters in liver and 8 in muscle (plus one altered by CR in the opposite directions in the two phenotypes). We suggest that these steps of insulin signaling are involved in the control of whole animal insulin sensitivity and mammalian longevity.

## Materials and Methods

### Animals

GHRKO and normal mice were produced in the breeding colony at SIU-SOM Springfield, IL which was developed from mice kindly provided by J. J. Kopchick (Ohio University, Athens). Phenotypically normal siblings of GHRKO mice served as controls in these studies. Animals were weaned at 3 weeks of age and placed on Lab Diet Formula 5001 (Ralston Purina, St. Louis, MO). Animals were housed at 20–23°C on a 12/12 hour light/dark cycle. Sentinel animals were sent for serological testing every 3 months and the results were uniformly negative. These studies were approved by the Laboratory Animal Use and Care Committee of SIU-SOM.

### Longevity Study

The every other day (EOD) feeding paradigm was conducted in normal and GHRKO mice starting at approximately 8 weeks of age. Mice were gradually shifted to EOD by placing them on every third day fast for the first week and then EOD feeding throughout the remainder of the study. The survival of male mice used in this study (approximately 15–20 per phenotype/dietary treatment) was evaluated once all four groups reached median lifespan. At the time of analysis, the remaining survivors from this still ongoing study were 6% of the N AL, 43% of the N CR, 41% of the KO AL and 46% of the KO CR mice. Log-rank analysis for partial survivorship was conducted. At the time of analysis, all female treatment groups did not yet reach median lifespan. Animals in the longevity study were checked daily for health and survival, and were handled only for cage changes and bi-weekly body measurements. Animals that appeared near death (listless, unable to walk, and cold to the touch) or had large bleeding neoplastic growth approaching 10% of their body weight were euthanized and date of euthanasia was considered date of death.

### Metabolic Parameters

In the mice on the terminal insulin stimulation study, metabolic parameters were evaluated from blood collected from the orbital plexus after 10 months of 30% CR. Following a 12 hour fast, animals were anesthetized using isoflurane (Abbott Laboratories, Chicago, IL) and glucose levels were determined using a glucometer (Lifescan, Johnson & Johnson, New Brunswick, NJ.) and insulin levels were determined using an enzyme-linked immunosorbant assay (ELISA, Crystal Chem. Inc., Downers Grove, IL). Homeostatic Model of Assessment (HOMA) score was calculated as 22.5/(insulin [mU/L] X glucose [mmol/L].

### Insulin Stimulation Study

GHRKO mice and phenotypically normal male siblings were gradually calorie restricted starting at 8 weeks of age, by receiving 90% of the amount of food consumed by AL controls in the initial week, 80% the following week, and 70% for the remainder of the study. After one year of 30% CR, mice from all 4 groups (N AL, N CR, KO AL, and KO CR, n = 15–18 per group) were anesthetized [ketamine (100 mg/ml):xylazine (20 mg/ml), at a 0.1 ml per 10 grams of body weight] and injected in the inferior vena cava with either 10 IU/kg of porcine insulin (Sigma, St. Louis, MO) or with saline (control). Liver and hind limb muscle tissues were extracted and snap frozen at 1 and 3 minutes, respectively, after injection.

### Protein and Phosphoprotein Determination

After storage at −80°C, liver and muscle tissues in T-Per (Pierce, Rockford, IL) with phosphatase inhibitor (Pierce, Rockford, IL) and protease inhibitors (Sigma, St. Louis, MO) at approximately 1 ml per 1 g of tissue. ELISA for insulin (CrystalChem, Downers Grove, IL), IR, IR pY1158, IRS-1, IRS-1 pS312, AKT1 and AKT1 pS473 were used for quantification of cellular proteins in accordance with manufacturer's instructions (Biosource Camarillo, CA).

For immunoprecipitation (IP), equal amounts of solubilized protein were incubated at 4°C overnight with ∼4ug/ml of specific antibody. Polypeptide-Immuneglobin complexes were then collected by incubation with protein A-sepharose beads (Sigma, St. Louis, MO) washed solubilization buffer A, and boiled in Laemmli sample buffer (Biorad, Hercules, CA). Antibodies (Ab) against pan p85, AKT2, AKT (pS473), mTOR, mTOR (pS2448), and GLUT4 (Cell Signaling Technology, Inc. Danvers, MA) were used according to manufacturer's suggestions. Non-specific IRS Tyr phosphorylation of p85 was determined by detecting anti-pY99 (Santa Cruz Biotechnology, Santa Cruz, CA) signal in ∼180 kDa region in the anti-pan p85 immunoprecipitates.

Immunoblotting was performed according to standard protocol. Protein content in tissue homogenates extracted with T-Per (described above) was determined by the BCA protein assay (Pierce, Rockford, IL). Protein lysates (40–60 ug) were subjected to SDS-PAGE using Criterion XT Precast Gels (BioRad, Hercules, CA), transferred to nitrocellulose membranes (BioRad, Hercules, CA) and even loading was verified using MemCode Reversible Protein Stain Kit (Pierce, Rockford, IL). Membranes were blocked for 1 hour at room temperature with either 5% dry skim milk or 3% BSA when determining phosphorylated proteins, in TBST (TBS+0.05% Tween-20). Blots were then washed with TBST and incubated with the primary Ab diluted in the appropriate Ab-specific blocking solution suggested by the manufacturer. ECL Plus chemiluminescent reagent was used for immunodetection (G.E. Healthcare Bio-sciences Corp, Piscataway, NJ). Digital images of blots were captured using a CCD camera (Hitachi Genetic Systems, Ameda, CA) and quantified using GeneTools software (SynGene, Cambridge, England).

### Statistical analysis

Kaplan-Meier survival curves were used for survival analysis using log-rank test to evaluate significance of survivorship between groups. Median lifespan represents the age at which 50% of the population within groups remained alive and was reported with the corresponding hazard ratio (HR) and confidence interval (CI). Analysis of phenotype X diet was used to reveal interactions of characterization factors upon the phenotype under analysis, with subsequent independent Student's t-tests for within group comparisons. Analysis of basal and insulin-stimulated protein concentration across all groups was analyzed with three-way Analysis of Variance (ANOVA) followed by subsequent two-way ANOVA's and Students t-tests within groups when warranted. All statistics were conducted using SPSS version 13.0 (SPSS, Chicago, IL) with α = 0.05. All graphs were made using Prism 4.02 (GraphPad Software, San Diego CA.). Alpha is set to 0.05. With the exception of longevity data, all values are reported as mean±Standard Error of the Mean (SEM) throughout the figures and text.
